RETRACTED

# Oleuropein Improves Cognitive Dysfunction and Neuroinflammation in Diabetic Rats through the PI3K/Akt/mTOR Pathway

**DOI:** 10.1155/2022/5892463

**Published:** 2022-04-28

**Authors:** Jianru Shang, Shan Che, Mingjie Zhu

**Affiliations:** ^1^Department of Critical Care Medicine, Renmin Hospital, Hubei University of Medicine, Shiyan Hubei 442000, China; ^2^Department of Ultrasound, Renmin Hospital, Hubei University of Medicine, Shiyan Hubei 442000, China; ^3^Department of Endocrinology, Renmin Hospital, Hubei University of Medicine, Shiyan Hubei 442000, China

## Abstract

**Objective:**

To explore the effect and mechanism of oleuropein on cognitive dysfunction and neuroinflammation in diabetic rats.

**Method:**

A diabetic rat model was constructed using streptozotocin, and the diabetic rats were divided into 3 groups with different treatment for 4 weeks, named STZ group (gavaged with normal saline), STZ+LOE group (40 mg/kg oleuropein, and STZ+SITA group (30 mg/kg sitagliptin). The fasting blood glucose (FBG), fasting serum insulin levels, and HOMA-IR index were measured in rats. After the last treatment, the Morris water maze experiment was carried out, and the rats were first subjected to training experiments for 4 consecutive days; the escape latency, number of crossing platform quadrant intersections, time spent in the target quadrant, and swimming speed were recorded. Additionally, the malondialdehyde (MDA), myeloperoxidase (MPO) content, superoxide dismutase (SOD) activity, interleukin- (IL-) 1*β*, tumor necrosis factor (TNF-*α*), and phosphatidylinositol 3-kinases (PI3K)/threonine-protein kinase (Akt)/mTOR expression levels in rat hippocampus tissues were detected.

**Results:**

Oleuropein reduced insulin resistance, spatial learning, and memory ability in diabetic rats. It also could improve oxidative stress and inflammatory response and activate the PI3K/Akt/mTOR signaling pathway in hippocampus tissues.

**Conclusion:**

Oleuropein ameliorates cognitive dysfunction and neuroinflammation in diabetic rats by regulating the PI3K/Akt/mTOR signaling pathway.

## 1. Introduction

Diabetes mellitus (DM) seriously affects people's health. In the past 10 years, the number of diabetic patients worldwide has almost doubled, and it is estimated to reach 669 million by 2045 [1]. DM is a metabolic disease induced by various etiologies, characterized by chronic hyperglycemia. Type 2 diabetes mellitus (T2DM) is the most prevalent subtype of DM, accounting for approximately 90% to 95% of the total DM cases [2]. Existing studies have reported that DM can lead to various complications, including diabetic retinopathy, diabetic nephropathy, cognitive dysfunction, and neuroinflammation [3]. Among the complications, cognitive dysfunction is a common one; according to statistics, the overall prevalence of dementia and cognitive impairment is 13.1% in diabetic patients aged 65-74 years and 24.2% in those aged 75 years and above [4]. In addition, studies have shown that patients with type 1 diabetes have a 65% increase in the risk of dementia, while T2DM patients have a 37% increase [5]. Neuroinflammation is a major risk factor for cognitive impairment and can be induced by DM [6]. Hyperglycemia caused by T2DM leads to increased mitochondrial respiration in endothelial cells, pericytes, and astrocytes, promoting the production of reactive oxygen species (ROS) and oxidative stress. Enhanced ROS activates NF-*κ*B, AP-1, and STAT pathways and in turn results in upregulation of inflammatory cytokines. ROS also can interfere with astrocyte communication by inhibiting the folding of the connexins. Astrocyte damage can be improved by using antioxidants and chaperone proteins. ROS-caused damage ultimately leads to loss of pericytes and breakdown of the blood-brain barrier, and such damage, if left untreated, can result in cognitive impairment [7].

RETRACTED

There is no clinically effective treatment for cognitive impairment and neuroinflammation in diabetic patients, although many attempts have been made. For example, some studies have tried to control blood glucose in T2DM patients, which can reduce the rate of brain atrophy but cannot improve cognitive dysfunction [8]. By contrast, intranasal insulin treatment has been proved to improve cognitive impairment in type 1 diabetic patients; such treatment reduces intracellular amyloid plaques and promotes tau protein phosphorylation, thereby stabilizing microtubules and enhancing tubulin polymerization [9]. In addition, many studies have focused on the treatment of cognitive impairment with diabetes drugs and have found that glucagon-like peptide-1 mimetic drugs are resistant to protease cleavage and can affect key pathophysiological pathways, thus preventing the development of DM and memory impairment [10]. Although these drugs can promote insulin release from the pancreas, they are limited by their short half-life [10]. Therefore, it is necessary to find new drugs for DM-induced cognitive dysfunction. Oleuropein is a phenolic compound abundant in olive [11]. Recent preclinical and clinical studies have identified the therapeutic effects of oleuropein on various human diseases. For example, Al-Azzawie and Alhamdani found that oleuropein was effective in the treatment of DM [12], and Moosmann and Behl demonstrated that oleuropein had neuroprotective effects [13]. It can be seen that oleuropein exhibits beneficial biological and pharmacological effects on humans, but there is no relevant research on its effects on cognitive dysfunction and neuroinflammation in diabetic patients. Therefore, this paper explores this unsolved question using a rat model of DM, aiming to find new ideas and provide certain experimental data for the clinical treatment of DM.

RETRACTED

## 2. Materials and Methods

### 2.1. Construction and Treatment of Diabetic Rat Model

Twelve adult male SD rats weighing around 180-220 g were selected. Three rats were randomly chosen as the control group and were fed with normal diet. The remaining 9 rats were used to establish T2DM model. The rats were fed with a high-fat and high-sugar diet for 4 weeks, and then, 35 mg/kg streptozotocin (STZ) was intraperitoneally injected; after 72 h, the rats with fasting blood glucose (FBG) > 13.9 mmol/L and the random blood glucose >16.7 mmol/L were considered as diabetic rats. Subsequently, rats in each group were treated differently. For rats in the control group, the same amount of sodium citrate buffer was injected intraperitoneally. For the rats with successful modeling, they were intragastrically administered with the same amount of saline, 40 mg/kg oleuropein, and 30 mg/kg of sitagliptin, and named STZ group, STZ+OLE group, and STZ+SITA group, respectively. The rats in each group were gavaged once a day for 4 weeks. After treatment, the rats were euthanized to collect their brain tissue. The animal experiments described in this study were authorized by the Experimental Animal Ethics Committee of Guangdong Medical Experimental Center.

### 2.2. Fasting Blood Glucose Test

After the start of treatment, fasting blood glucose of the rats in the control group, STZ group, STZ+OLE group, and STZ+SITA group was measured every week. All rats fasted for 12 h before the test but were given free access to water. Subsequently, the rats were fixed, and 1/4 of the end of the tail was disinfected with alcohol cotton balls and was then punctured with a blood lancet to take an appropriate amount of blood. The blood was dropped onto the test area of the blood glucose test strip, and the strip was then immediately read by the ACCU-CHEK blood glucose meter (Roche Diagnostics, Shanghai, China).

### 2.3. Detection of Fasting Serum Insulin Levels

At the end of the experiment, the venous blood of the rats in each group was collected through the tail vein and centrifuged at 2000 rpm for 20 min at 4°C. The supernatant transferred to a new centrifuge tube was serum. The serum insulin levels of rats in each group were measured in strict accordance with the instructions of the insulin ELISA assay kit (MLBIO, Shanghai, China).

RETRACTED

### 2.4. Calculation of HOMA-IR Index

At the end of the experiment, FBG value and fasting serum insulin level of rats in each group were detected to calculate the HOMA-IR index (HOMA − IR = (FBG value × serum insulin level)/22.5).

### 2.5. Morris Water Maze Experiment

The Morris water maze (Yuyan Instruments, Shanghai, China) was a circular pool with a white inner wall, 150 cm in diameter, and 50 cm in height. The pool was divided into 4 quadrants labeled with different markers. After the last treatment, the rats were subjected to a training experiment for 4 consecutive days. Adaptive training was to place the rats in a water maze without a platform and allow them to swim freely for 120 s. On completion of the training, they were taken out to wipe them dry, so as to reduce the influence of grasping and water environment. Then, a navigation test was performed. Specifically, the rats were randomly placed in 1 quadrant and faced the pool wall, and the time it took to find the platform (escape latency) was recorded. The timer was stopped 10 s after reaching the platform. If the rat did not find the platform within 120 s, they were led to the platform, left on it for 10 s, and taken out. The navigation test was carried out once in the morning and once in the afternoon for 5 consecutive days. Finally, a formal experiment was conducted to evaluate the spatial learning and memory ability of the rats. Escape latency, number of crossing platform quadrant intersections, time spent in the target quadrant, and swimming speed were all recorded.

### 2.6. Biochemical Detection

Hippocampal tissue was isolated from 50 mg of brain tissue, and then, RIPA lysis buffer was added (ThermoFisher, Waltham, MA, USA). After full homogenization, the tissue was centrifuged at 12000 rpm for 30 min at 4°C and the supernatant was taken. The levels of malondialdehyde (MDA), myeloperoxidase (MPO), and superoxide dismutase (SOD) activity in the tissue were detected by the AU-400 automatic biochemical analyzer (Olympus, Tokyo, Japan).

### 2.7. ELISA Detection

The same homogenization method as Section 2.6 was used to obtain the hippocampal tissue. The levels of IL-1*β* and TNF-*α* in the hippocampus of rats in each group were detected in strict accordance with the instructions of ELISA kits of IL-1*β* (BLKW Biotechnology, Beijing, China) and TNF-*α* (Xitang Bio, Shanghai, China).

### 2.8. Western Blot

First RIPA buffer was adopted to extract total protein from 50 mg of hippocampal tissue. The obtained protein was then centrifuged at 12,000 rpm for 30 min at 4°C, and the supernatant was taken as the total protein. Protein concentrations were determined using the BCA assay (ThermoFisher). Then, 20 *μ*g of protein was separated on a 10% SDS-PAGE and transferred to a polyvinylidene fluoride (PVDF) membrane. The membrane was blocked with 5% skim milk for 1 h, followed by overnight coculture of primary antibodies of anti-rat phosphatidylinositol 3-kinase (PI3K), phosphorylated (p)-PI3K, Akt, p-Akt, mTOR, p-mTOR, or *β*-actin (all purchased from Abcam, Cambridge, United Kingdom) at 4°C. After that, the membrane was incubated with the corresponding secondary antibodies (Abeam) for 1 h at room temperature. After labeling with the Chemiluminescent (ECL) Substrate Kit (Yan Hui Bio, Shanghai, China), ECL imaging system JP-K300 was used to scan immunoblot bands (GeeBio (Jinpeng), Shanghai, China), with *β*-actin as an internal reference for whole-cell or cytoplasmic proteins. Gray-scale values were analyzed with Image Lab™ software.

RETRACTED

### 2.9. Statistics Analysis

SPSS 26.0 (IBM-SPSS, Chicago, IL, USA) was used for multiple comparisons using LSD test; with a/b/c indicating the difference between groups, the same superscript suggested no significant difference (*p* > 0.05) and different superscripts a significant difference (*p* < 0.05). *T*-test was used for comparison between the two groups, with *p* < 0.05 as a cut-off value of statistical significance. The results were expressed as mean ± standard error (mean ± SE).

## 3. Results

### 3.1. Oleuropein Can Reduce Fasting Blood Glucose and Improve Insulin Resistance in Diabetic Rats

The blood glucose analysis showed that the FBG levels of the rats in the control group were always within the normal range, while that in the STZ group remained at a high level (>16.7 mmol/L). The FBG level of rats in the STZ+OLE and STZ+SITA groups was high before treatment, but with the increase of treatment time, the level showed a downward trend (Figure 1(a), *p* < 0.05). After 4 weeks of treatment, compared with the STZ group, the FBG of the STZ+OLE group, and STZ+SITA group significantly decreased, and there was no significant difference between the STZ+OLE group and STZ+SITA group. Compared with the control group, the fasting serum insulin levels and HOMA-IR index of the other 3 groups were significantly increased. However, compared to the STZ group, the levels of these two indexes showed a significant decrease after oleuropein and sitagliptin (*p* < 0.05), and no marked differences between the STZ+OLE group and the STZ+SITA group (Figures 1(b) and 1(c)).

### 3.2. Oleuropein Improves Spatial Learning and Memory in Diabetic Rats

The Morris water maze test results showed that on the first day, the escape latency of rats in the control group was significantly lower than in the other 3 groups (*p* < 0.05), and there was no statistically significant difference among the STZ group, STZ+OLE group, and STZ+SITA group (*p* > 0.05). With the increase of training time, the escape latency of the rats in each group gradually decreased, but that in the STZ group was always significantly longer than the control group (*p* < 0.05). From the 3^rd^ day, the escape latency in the STZ+OLE group and STZ+SITA group was significantly lower than that of the STZ group (*p* < 0.05) (Figures 2(a) and 2(b)). Compared with the control group, a significant reduction in the number of crossing intersections in the platform quadrant and the time spent in the target quadrant was found in the other 3 groups (*p* < 0.05); compared with the STZ group, treatment of oleuropein and sitagliptin led to higher levels of these two measures (*p* < 0.05) (Figure 2(c)). Additionally, streptozotocin treatment caused a decrease of the average swimming speed of the rats, but the difference was not statistically significant (*p* > 0.05) (Figure 2(d)).

RETRACTED

### 3.3. Oleuropein Reduces Oxidative Stress in Hippocampus Tissue of Diabetic Rats

The detection results of blood biochemical indicators showed that streptozotocin induced a marked increase of the contents of MDA and MPO and a decrease of SOD activity (*p* < 0.05). Compared with STZ group, STZ+OLE group and STZ+SITA group presented significantly decreased contents of MDA and MPO and increased SOD activity in the hippocampus tissue (*p* < 0.05), and no significant difference was identified in the latter two groups (Figure 3).

### 3.4. Oleuropein Attenuates Neuroinflammation in Diabetic Rats

The results of ELISA detection of inflammatory factors in hippocampal tissue samples showed that the levels of IL-1*β* and TNF-*α* in the hippocampus tissue were significantly increased after streptozotocin treatment (*p* < 0.05), but their levels decreased markedly after treatment with oleuropein and sitagliptin (*p* < 0.05, Figure 4). And the difference between the STZ+OLE group and the STZ+SITA group was not statistically significant (*p* > 0.05).

### 3.5. Oleuropein Activates the PI3K/Akt/mTOR Signaling Pathway in Hippocampus Tissue of Diabetic Rats

Western blot analysis of key proteins of the PI3K/Akt/mTOR signaling pathway in rat hippocampus tissue showed that compared with the control group, the expression levels of p-PI3K, p-Akt, and p-mTOR and the ratios of phosphorylation (p-PI3K/PI3K, p-Akt/Akt, and p-mTOR/mTOR) in hippocampal tissues of the other 3 groups decreased significantly (*p* < 0.05). Compared with the STZ group, the expression levels of p-PI3K, p-Akt, and p-mTOR in hippocampal tissues of rats treated with oleuropein and sitagliptin were significantly increased, and the ratios of phosphorylation (p-PI3K/PI3K, p-Akt/Akt, p-mTOR/mTOR) were significantly increased (*p* < 0.05) (Figure 5).

RETRACTED

## 4. Discussion

The two main forms of DM are type 1 diabetes and type 2 diabetes [14]. The global prevalence of DM among people over the age of 65 is 18.8%. In 2017, the number of diabetic patients aged 65-99 was estimated to be 122.8 million [15] and approximately 171 million cases in global population. Cognitive dysfunction is an important complication of diabetes. Clinical studies and animal evidence prove that people with diabetes are at a higher risk of developing behavioral disorders manifested as cognitive deficits and even dementia [16]. In addition, some studies have shown that there is a direct relationship between neuroinflammation and cognitive dysfunction, and proinflammatory cytokines have been considered as key factors in the progression of cognitive dysfunction [17]. At present, many antidiabetic drugs have been used clinically to treat DM. However, existing antidiabetic drugs are ineffective for their complications [18], including cognitive impairment, and even have had gastrointestinal side effects, such as nausea, vomiting, diarrhea, and lactic acidosis [19]. Therefore, there is a need to find a natural-derived drug with good curative effects and few side effects for the treatment of diabetes.

In recent years, oleuropein, a polyphenolic compound rich in olive oil and olive tree leaves, has attracted the scientific community's attention for its various reported health benefits. Oleuropein is known for its blood pressure-lowering effects; it can reduce systolic and diastolic blood pressure in animal models when administered via intraperitoneal or intravenous injection [20]. Additionally, oleuropein has been shown to have cardioprotective, anti-inflammatory, antioxidant, anticancer, antiangiogenic, and neuroprotective functions [21]. Thus, it may have therapeutic potential for a variety of human diseases. In the results of this study, oleuropein significantly reduced FBG levels in diabetic rats and improved insulin resistance. Similarly, a study demonstrated that treatment with oleuropein in a streptozotocin-induced diabetic animal model improved hyperglycemia, significantly reduced FBG level, glycated hemoglobin (HbA1c), and improved glucose tolerance [22]. Another study showed that oleuropein inhibited the activity of glucose-6-phosphatase in the liver, increased serum insulin, and enhanced the antioxidant activity of pancreatic tissue by increasing the glucose uptake in the isolated psoas major muscles [23]. A moderate lethal dose of oleuropein has not been established in acute toxicity studies, because no side effects or lethal conditions have been observed in mice even at doses up to 1000 mg/kg [24]. Clinical studies assess the effect of oleuropein on blood glucose management using a variety of markers, including plasma glucose peaks, dipeptidyl peptidase 4 (DPP-4) activity, glucagon-like peptide-1, insulin secretion, and *β*-cell reactivity, and suggest oleuropein also has antidiabetic effects in humans [25]. Collectively, oleuropein is an effective and safe drug for the treatment of diabetes.

RETRACTED

Oleuropein is a multifunctional active substance, and its multiple pharmacological features were attributed to its powerful antioxidant effects [26]. Previous studies indicated that oleuropein could chelate metal ions, such as Cu^2+^ and Fe^2+^, and slow down free radical generation. Both oleuropein and its metabolite hydroxytyrosol have the optimal structure for antioxidant and scavenging activities [27]. In Alirezaei et al.'s experiments, it was shown that oleuropein could act as an antioxidant to improve spatial memory impairment in rats [28]. Other research groups have confirmed that olive leaf extract reduces age-induced oxidative stress in major organs of aged rats [29]. Oleuropein treatment after spinal cord injury has neuroprotective effects in rats [30]. In our study, oleuropein also improved spatial learning and memory ability in diabetic rats. Nasrallah et al. conducted experiments in rats with renal ischemia-reperfusion injury and found that oleuropein significantly reduced the expression of AMP-activated protein kinase, endothelial nitric oxidase-related oxidative stress protein, and at the same time reduced inflammatory proteins and apoptosis proteins, suggesting that oleuropein can be used as a therapeutic agent to slow renal ischemia-reperfusion injury through its antioxidant, anti-inflammatory, and antiapoptotic properties [31]. Our results demonstrated that oleuropein significantly decreased the content of MDA and MPO, significantly increased the activity of SOD, and significantly reduced the levels of IL-1*β* and TNF-*α*. Collectively, oleuropein can protect the hippocampal tissue of rats by decreasing oxidative stress and inflammatory response.

It is well known that the PI3K/Akt/mTOR signaling pathway is closely related to the occurrence of oxidative stress and inflammatory response. Huang et al. found that aflatoxin B 1 caused severe damage to testicular development and spermatogenesis because aflatoxin B inhibited the PI3K/AKT/mTOR signaling pathway related to oxidative stress [32]. In addition, regulating the PI3K/Akt/mTOR signaling pathway can achieve inhibition of oxidative stress and inflammatory responses and alleviation of lipopolysaccharide-induced acute lung injury in mice [33]. The PI3K/AKT/mTOR pathway plays a key role in autophagy and inflammation: PI3K is a class of lipid kinases, and AKT is the central mediator of the PI3K pathway. After activation of PI3K, the phosphorylation of AKT can further phosphorylate the downstream mTOR and other target proteins, thereby mediating various biological effects such as inflammation, autophagy, and apoptosis. The PI3K/Akt signaling pathway is involved in the regulation of proinflammatory gene-stimulated NF-*κ*B activity. Akt can regulate the activity of transcription factors including NF-*κ*B. When endotoxin and TNF-*α* stimulate monocytes/macrophages, activation of the AKT pathway can inhibit the NF-*κ*B translocation and reduce the further activation of monocytes/macrophages to reduce the secretion of inflammatory cytokines. According to our study, oleuropein activated the PI3K/Akt/mTOR signaling pathway in hippocampus tissues of diabetic rats. Thus, it can be explained that oleuropein exerts its pharmacological function by regulating the PI3K/Akt/mTOR signaling pathway.

RETRACTED

## 5. Conclusion

Oleuropein regulates the PI3K/Akt/mTOR signaling pathway to ameliorate oxidative stress and inflammation in hippocampal tissue and improve cognitive dysfunction, neuroinflammation, and insulin resistance in diabetic rats. Oleuropein has the potential to be a therapeutic drug for the treatment of diabetes-induced cognitive dysfunction and neuroinflammation. However, this test has only performed on rats, so further clinical trials are needed to provide more exact experimental data for the clinical application of oleuropein.

## Figures and Tables

**Figure 1:** The effect of oleuropein on insulin resistance in diabetic rats. (a) Fasting blood glucose levels during the test period (0-28 days). (b and c) At the end of the experiment (the 28th day), the fasting insulin levels (b) and HOMA-IR index (c). Each set contains data from 3 samples tested independently; LSD test was used for multiple comparisons. ^∗∗^*p* < 0.05 vs. control group and ^##^*p* < 0.05 vs. STZ group.

**Figure 2:** Effects of oleuropein on spatial learning and memory in diabetic rats. (a) The escape latency of rats in the Morris water maze on days 1, 2, 3, and 4. (b) The number of crossing intersections of the platform quadrant in Morris water maze test. (c) The time spent by rats in the target quadrant in the Morris water maze test. (d) The swimming speed of the rat in the Morris water maze test. Each set contains data from 3 samples tested independently; LSD test was used for multiple comparisons. ^∗∗^*p* < 0.05 vs. control group and ^##^*p* < 0.05 vs. STZ group.

RETRACTED

**Figure 3:** The effect of oleuropein on oxidative stress in the hippocampus tissue of diabetic rats. Blood biochemical analysis showed MDA (a), MPD (b), and SOD (c) levels in hippocampus tissue of rats in each group. MDA: malondialdehyde; MPO: myeloperoxidase; SOD: superoxide dismutase. Each set contains data from 3 samples tested independently; LSD test was used for multiple comparisons. ^∗∗^*p* < 0.05 vs. control group and ^##^*p* < 0.05 vs. STZ group.

**Figure 4:** The effect of oleuropein on neuroinflammation in diabetic rats. ELISA analysis of inflammatory factors including IL-1*β* (a), and TNF-*α* (b) in the hippocampus tissue of the rats. Each set contains data from 3 samples tested independently; LSD test was used for multiple comparisons. ^∗∗^*p* < 0.05 vs. control group and ^##^*p* < 0.05 vs. STZ group.

**Figure 5:** The effect of oleuropein on the PI3K/Akt/mTOR signaling pathway in hippocampus tissue of diabetic rats. Western blot original images (a) and quantitative gray-scale analysis (b) of PI3K/Akt/mTOR signaling pathway-related proteins in the hippocampus tissues of rats. Each set contains data from 3 samples tested independently; LSD test was used for multiple comparisons. ^∗∗^*p* < 0.05 vs. control group and ^##^*p* < 0.05 vs. STZ group.

## Data Availability

The data used to support the findings of this study are available from the corresponding author upon request.
